# Machine Learning and IoT-Based Waste Management Model

This article has been retracted.

**DOI:** 10.1155/2021/5942574

**Published:** 2021-08-26

**Authors:** Rijwan Khan, Santosh Kumar, Akhilesh Kumar Srivastava, Niharika Dhingra, Mahima Gupta, Neha Bhati, Pallavi Kumari

**Affiliations:** ^1^Department of Computer Science and Engineering, ABES Institute of Technology, Ghaziabad, U.P., India; ^2^Department of Mathematics, College of Natural and Applied Sciences, University of Dar es Salaam, Dar es Salaam, Tanzania; ^3^Department of Computer Science and Engineering, ABES Engineering College, Ghaziabad, India

## Abstract

A rapid rise in inhabitants across the globe has led to the inadmissible management of waste in various countries, giving rise to various health issues and environmental pollution. The waste-collecting trucks collect waste just once or twice in seven days. Due to improper waste collection practices, the waste in the dustbin is spread on the streets. Thus, to defeat this situation, an efficient solution for smart and effective waste management using machine learning (ML) and the Internet of Things (IoT) is proposed in this paper. In the proposed solution, the authors have used an Arduino UNO microcontroller, ultrasonic sensor, and moisture sensor. Using image processing, one can measure the waste index of a particular dumping ground. A hardware prototype is also developed for the proposed framework. Thus, the presented solution for the efficient management of waste accomplishes the aim of establishing clean and pollution-free cities.

## 1. Introduction

The waste management system predominantly corroborates the disposal and treatment of different types of waste. Thus, it safeguards human beings, animals, and surroundings [1]. Adequate waste management techniques can save much money, which will lead to improved air quality and less environmental pollution. Simultaneously, the advanced regions are discovering and implementing some efficient techniques for efficient waste management and coming up with enormous constructive results [2]. It will be impossible to manage such a huge amount of waste in the upcoming five years by the current situation. Thus, it is better to take all the necessary actions required for the effective management of waste. Therefore, we must adopt the best techniques and practices to treat waste efficiently to have healthy environment [3]. Worldwide, there is an enormous increase in the generation of waste per day. Approximately 1.9 billion tons of waste is generated annually, with a minimum of 35% that is not treated securely. As per the reports, the waste generated per person per day varies from 0.17 to 4.67 kilograms. The overall waste is anticipated to exceed about 45 billion tons by 2055, which will be over double growth for the identical period. Income and generation of waste are directly proportional to each other. Waste is a huge income source, so its treatment and disposal must be done in the best possible way. It is estimated that, by 2050, per day waste generation of the low-income and middle-income nations would rise to 45%, and for the high-income countries, it can increase to 20% [4].

The most effective solution to overcome the problem of environmental pollution is the use of the Internet of Things- (IoT-) and machine learning- (ML-) based waste management system [5]. These technologies can provide real-time information about the waste and provide an optimized path for the waste collection trucks, reducing the cost and time for the overall process. The issues faced by current waste management systems are improper scheduling; that is, the waste collectors do not know that they had to pick the waste. They also do not know precisely about the drop-off location [6]. One significant application is that IoT innovation has become an effective apparatus to manufacture brilliant urban communities. A fundamental issue for a smart city is the expansion of waste generation with quickened populace development in urban communities [7].

Waste management may be a daily task in metropolitan zones involving arranging waste truck routes in which natural, monetary, and social elements must be considered. Secondly, the length needs to be abbreviated to maintain a strategic distance from high fuel costs and diminish the work sum by applying the diagram hypothesis [8]. A couple of arrangements have presented IoT gadgets to appraise inboxes' fill levels and send this information over the web for better decisions. Waste management hierarchy is shown in Figure 1.

Although human interference is equally essential in collecting, transportation, and efficient waste disposal, the sensors are connected to the microcontroller [9]. Hence, they will provide real-time information regarding the dumping grounds' waste index and the level of waste of the dustbins. Due to the rapid rise in inhabitants worldwide, the usage of every material has also increased exponentially, and the amount of waste generated every day is also very large. The civic authorities' ordinary trash cans are also becoming a major reason for the inefficient collection and management of waste [10]. None can use smart bins in place of them, which will provide real-time information and reduce the cost and the time of waste collection. Lack of awareness among people is also creating hindrances in the efficient management of waste. The waste management system proposed in this paper will detect the waste level in the dustbins and the dumping grounds' waste index. In this system, the authors used the Arduino UNO microcontroller. Sensors are connected with the microcontroller for processing. Here, we have deployed an ultrasonic sensor and moisture sensor. The ultrasonic sensor will depict the assorted distance from waste in the dustbins. Essentially, it is used for the space measurement purpose and the moisture sensor determines whether the waste is moist or dry. Using image processing, we will measure the waste index of a specific dumping ground. The waste index is often low, medium, or high. Accurate categorization of waste is completed by using a neural network. A dumper truck database has been generated in the given system so that data and details of dumper truck ID, meeting date, meeting time of garbage collection, and so on are collected. The mobile application developed by us will monitor important time movement and track vehicular movement. It will send an optimized track to destination waste to the teamster. The authors employ integrated software and hardware modules.

In this paper, the authors developed a prototype for smart waste management system using machine learning- and IoT-based techniques. The 4 most important parts in this paper include (a) literature review, (b) waste management problem in smart cities, (c) proposed system and hardware parts used for prototype system, and (d) comparison of prototype with other systems and conclusion.

## 2. Literature Review

Waste management is an essential part of maintaining a city's hygiene and health. Developed countries now have adequate resources and equipment to sustain these favorable conditions, such as up-to-date and even real-time waste generation statistics, qualified personnel, and current fleets of collection trucks equipped with the most cutting-edge technical breakthroughs or instruments, such as geographical information systems. Finally, collection routes and the number of trucks required for each waste proportion in each region were estimated. All of this activities contribute to the solution of the waste disposal problem in a single zone where immediate solutions are required to advance toward sustainable development [11]. However, these garbage collecting methods have contributed to sustainability by reducing trash, pollution, and expenses while also enhancing the quality of recovered garbage. Thus, industrialized economies should take note of how trash collection methods have affected resource recovery. The construction of buy-back centers should be prioritized in emerging nations, where the majority of garbage is retrieved informally. The influence of buy-back centers on resource recovery should be examined in a future study on establishing recovery programs in emerging countries. The quantity of reusable, recyclable, and remanufactured garbage collected from the informal waste sector should be factored in [12].

As a result of the curbside component in the preimplemented system, the mixed collection system has more excellent material separation rates, better recycling rates, and lower contamination rates than the exclusive drop-off system [13]. Furthermore, attempts to reduce waste had a substantial impact on just recycling behavior. However, attitudes toward resource efficiency had a negligible impact on all waste management behaviors, indicating that individuals in the European Union (EU) are unaware of the link between waste reduction and resource efficiency [14]. The transportation of garbage (typically over long distances and with high frequency) to large processing facilities and the complicated waste separation systems necessary are the weakest points of centralized waste management systems. Both consume much energy and contribute to the worsening of climate change. Garbage treatment in homes allows for the elimination of the inconvenient nature of extended waste management systems. Several waste management techniques may be used at home, depending on the amount of space, time, and financial resources available to the householders. Unfortunately, most of them (composting, anaerobic digestion, and open burning) can only handle organic waste. Composting is the most frequent waste management technology at the household level. There are various processes and types of equipment available, ranging from simple homemade boxes to more advanced but more expensive automated composters. Composting allows the nutrients in the biomass to be returned to the soil. Consumers can get high-quality fertilizer. It will, however, take time. Furthermore, microbes use the energy present in the waste. It is lost from the standpoint of residents [15].

The system designed in this research is based on a prototype of IoT sensing. It monitors the garbage level in the garbage bins and sends the data to a server for storage and processing (through the Internet). This information is used to calculate the best collecting routes for the personnel. We would aim to improve the system in the future for diverse types of garbage, such as solid and liquid wastes [16]. The smart garbage bins are monitored in real time by the IoT-based garbage collection system [17, 18]. It allows a user to keep track of the garbage bins' fill level, fill status, volatile organic compounds (VOC) level, temperature, and humidity from anywhere at any time. It also identifies which garbage containers should be emptied at the end of each collection cycle. In addition, the navigation system suggests the best driving routes for collecting rubbish from the designated containers. The technology reduces travel distance significantly as compared to the previous approach, resulting in a more efficient garbage collecting procedure and lower costs [19]. Finally, the authors think that their work has contributed to waste management since it is a valuable tool for technical personnel who may develop and enhance a town's garbage collecting system [20–22]. The authors suggested a unique municipal solid waste (MSW) collection optimization model based on the actual real-world trash-collecting scenario in Sfax and then used the new innovative routing method for MSW collection. Throughout the study, all of the approaches have been explicitly presented [23].

In a previous research, an optimum path planning algorithm based on an ILP (integer linear programming) was provided, with the capacity of simultaneously choosing the number of trucks to utilize and their ideal routes, as well as the ability to take into account limits such as acoustic effect in the streets or maximum route lengths for each truck. The technique is integrated into the open-source Net2Plan-GIS planning tool, which makes it easier to apply it in real-world scenarios by enabling data from Geographic Information System (GIS) databases to be entered [24]. There is a review of the literature on facility location issues (FLPs). The study attempted to examine the underlying notions of the distance function, which are particularly significant in FLPs, in order to explain the notion of this class of issues. Because of the issues' complexity, numerous mathematical models were studied, and several optimization strategies have been applied to discover near-optimal solutions. The review continues by describing some important research in which FLPs are directly applied to rubbish collection, an essential waste management activity [25].

Designers can help to reduce building waste by prefabricated components, standardizing materials, and utilizing emerging Building Information Modeling (BIM) technology before physical building begins. The first step toward an efficient waste management plan is to design for limited waste. Water resources must be safeguarded and effectively managed across the world. Buildings play a critical role in wastewater reduction and water conservation efforts. Sustainable construction gives stakeholders the tools to increase efficiency and reduce waste and greenhouse gas (GHG) emissions [26]. The findings revealed that the respondents' knowledge, attitudes, and behaviors regarding food waste were all over the map. However, most respondents agree that minimizing food waste necessitates a systematic approach involving a cyclical process of reducing, reusing, and recycling to reduce the problem caused by poor food handling; hence, waste created during meal preparation is a concern in the home. Nonetheless, they largely agree with the advice that a mandatory food waste recycling system for private households is introduced immediately and then closely monitored by authorities in order to tackle the pressing issue of food waste efficiently and effectively [27].

Using convolutional neural network (CNN) to categorize the kind of e-waste and R-CNN to identify the category and size of waste equipment in photos, some studies proposed a unique way to photographic identification and classification of e-waste. The suggested system for capturing, uploading, and identifying photos in order to build a trash collection plan can also be used at municipal collection facilities that hold e-waste. In such instances, quicker R-CNN might identify more garbage equipment, as demonstrated in this study. Other types of equipment submitted for collection should be included in a future study to ensure that the categorization and detection systems are functional. This strategy might be extended to other bulky garbage categories with comparable garbage collecting issues [28]. The growing use of biobased goods has resulted in a slew of waste management concerns. First and foremost, it must be identified how these items are now managed, as these data are currently unavailable. Second, techniques for maximizing the value of biobased goods must be created [29]. It is worth noting that the approach has certain limitations in that the reviewers choose characteristics and features based on what they thought were essential for a study that focused on evaluating waste management strategies at the national level. A quantitative and analytical rating of IO models against a wider pool of parameters, for example, will enhance the review [30]. The future of waste management is a complex balancing act of diplomacy, technology, public access to information, and, most importantly, goodwill to improve the situation [31].

According to this report, the successful management of urban waste will be needed to fund MSW management. Municipal governments would be relieved of budgetary burdens if waste disposal reliability and resource recycling rates were improved. For example, collecting half of the MSW and recycling 15% of the plastic content will cover the expense of handling plastic-related waste; however, depending on the recovery rate, collection quality, and price of recovered plastic, the flow of financial resources can fluctuate. Additional policy initiatives, such as the standardization of packaging materials and infrastructure construction, will thus aid in the better management of MSW in the long run [32]. Only the financial and management aspects of Integrated and Sustainable Solid Waste Management (ISSWM) in Nepal are included in their report. In creating an ISSWM system for Nepalese municipalities, future studies may concentrate on other aspects, such as stakeholder desires, policy coherence, and household behavior [32].

The study authors suggested a scheme that demonstrates an intelligent way to capture waste in an intelligent environment. The device is based on an IoT sensing prototype that monitors bin waste levels and transmits the data to a server via Internet services. For further processing and analysis, the data processed on the server as well as in the cloud are used. Based on this information, the collecting area is divided into five areas, and four routes are built, each of which is allocated to a waste truck in order for it to reach the filled bins in the simulation successfully. The report concentrated on the system's performance and maintenance costs [33]. The authors demonstrated an intelligent waste management system that included sensors to track bin status [34, 35], the LoRa communication protocol for low-power, long-range data transmission, and TensorFlow-based object detection for waste recognition and classification. The model was able to detect and distinguish waste into metal, plastic, and paper categories. However, increasing the amount of training data, in this case, the number of waste images as well as the training time, increased the model's accuracy. Furthermore, for the purpose of upkeep, an automatic routing scheme may be created to define and locate the shortest path to the bin. With this in mind, the current waste management scheme will be strengthened, and society can benefit. With this in mind, the current waste disposal scheme should be changed, leading to a more environmentally friendly and healthy world [36].

The system proposed by the author is better than the existing system because the authors have used the concept of image processing to measure the waste index of a dumping ground which is not used in the existing system. This method of image processing is fast and effective. The solution mainly focuses on efficient waste collection processes. In this project, the authors have used image processing to find the waste index of a dumping ground. Waste index is waste per area. If the waste index of a particular dumping ground is high, then priority is given to that dumping ground. The authors have also deployed sensors in the dustbins which will help to find the priority of one dustbin over the other.

## 3. Waste Management Problem in Smart Cities

Management of waste is one of the biggest problems that is faced by the cities. Despite a considerable workforce of waste, such as waste collectors, scrap dealers and recyclers are involved in managing the waste in smart cities. The most affected section in the waste disposal system process includes the unrecognizing garbage collectors who form the country's largest informal sector. These waste collectors usually have their communities, which have 50–70 households, and all the family members are involved in collecting the waste across the country. These waste collectors manage approximately 15–20% of the city's waste, and all the members of their families are involved in this profession.

### 3.1. Lack of Awareness about Waste Management

Most people are not aware that inefficient waste collection and waste management can create environmental pollution. Due to a rapid rise in inhabitants across the globe in the last few decades, it is very difficult to manage such a huge amount of waste. We can spread awareness among common people by organizing workshops. The program is very important because it creates awareness among a country's citizens. Most people do not know about dry waste and wet waste in India, and they cannot differentiate between them. These people mainly belong to shanty town areas, so they do not know about segregation. To create attention about the sanitation, segregation of garbage in every city, and the community, organizing workshops and seminars regarding efficient waste management is very important. Spreading awareness among people will have a positive impact on efficient waste management.

### 3.2. Improper Classification of Municipal Waste

The improper classification and disposal of municipal waste can be very hazardous. It not only affects human and animal health but also can hinder the growth of plants. The only solution is proper classification, disposal, and treatment of municipal waste [37].

### 3.3. Participation of Organized Sector for Carrying Out Efficient Management of Waste

As the efficient waste management system's execution is becoming a necessity, the participation of people in that country in several practices for proper waste collection and disposal is also essential. We also see that the rag-picker who collects the garbage from the different areas of the cities or towns does not appreciate any reward from society. Therefore, giving the proper instruction to them is also very important. When every sector equally participates in managing waste, any country or city can become pollution-free [38].

### 3.4. Lack of Technical Solution and Public-Private Partnership

New technical solutions are essential for executing an effective waste management system, like the Internet of Things, machine learning-based technology, and some other new technologies. Some new technologies can prove to be the best in this field. So, there is a need for a public-private partnership for implementing this type of system that we found significantly less in the current scenario [39].

### 3.5. Transportation of Waste

Transportation is the main part which is used for managing the waste across the country. The collected waste is carried out using various vehicle types, such as trucks, tractors, and many more. In most of India's cities, there is a lack of transportation system and they may use some old vehicles that are not capable of carrying waste efficiently. These are the problems which are mainly faced in managing the waste. Proper and effective transportation can provide an optimized path, which saves a lot of time and money [40].

## 4. Proposed Method for Smart Waste Management

Waste collection and management is often discerning as a low-tech undertaking. However, IoT- and ML-based solutions have the power to transform individual waste containers into a web of smart, connected objects. A dumper truck database has been generated in the given system so that data and details of dumper truck ID, meeting date, meeting time of garbage collection, and so on are collected. This technique keeps track of all the truck driver's activities and the waste gathering system of waste management. This system allows on-time waste gathering and also allows automobile trace through database making use of Global Positioning System (GPS) automation.

The system proposed in Figure 2 by authors can administer and supervise the overall process of waste collection and efficient waste treatment and decrease the drawback such as usage of the minimal way, fuel price, cleansed nature, and available vehicle.

The Global Positioning System employs satellites to determine a vehicle, person, or other assets' precise position and records the asset's position at regular intervals. The trucks' details are then forwarded to the data centers with a remote correspondence interface. With the help of the tracking system, the authorities of a waste management organization can keep track of their vehicles. Our system provides an optimized path for collecting waste, which saves much time and increases the efficiency of the work done. In this system, we have used the Arduino UNO microcontroller. Sensors are connected with the microcontroller for processing. Ultrasonic sensor ranges from 2 cm to 400 cm measurement function of noncontact. Moisture sensors are also used to detect whether the waste is wet or dry. A mobile app is developed to store the history of the driver and various records related to waste. In this application, we also used image processing to measure the waste index of a particular dumping ground. The waste index can be low, medium, or high.

According to India's circumstances, the civic authorities are entirely accountable for properly managing different types of wastes in their particular metropolis. Still, the administration does not accomplish their duties to find efficient ways to collect, transport, and dispose of waste properly.

The real-time monitoring system is shown in Figure 3. Sometimes, the waste gets blended with excretory products of human beings and animals, which can spread many diseases. So proper and efficient management of waste becomes a necessity to have good hygiene. Segregation of waste at the source itself is an important strategy for the efficient management of waste. Waste segregation is not properly done in India. According to the latest reports, no country or city can achieve 100% segregation, but a maximum of 75% of segregation can be achieved with proper practices. The remaining 25% of waste remains in the environment. Proper segregation practices can lead to a healthy and hygienic environment.

## 5. Experimental Setup

Hardware components used are as follows:

- Arduino UNO microcontroller
- Ultrasonic sensor
- Moisture sensor buzzer
- LED
- Jumper wires

The smart waste management system can be administered and supervised using machine learning and the Internet of Things. The system proposed by the authors functions with the ultrasonic sensor and moisture sensor as shown in Figure 4. The ultrasonic sensor will depict the assorted distance from waste in the dustbins. This sensor ranges from 2 cm to 400 cm measurement function of noncontact. These sensors are deployed on the dustbins, and they detect the level of waste in the dustbins. The Arduino UNO microcontroller further gives the indications. Ultrasonic sensors provide the waste index (i.e., low, medium, or high) to the mobile application. This technique monitors the dustbins and notifies the level of waste in the dustbins. The system employs sensors, buzzer, Arduino UNO microcontroller, and LED. Therefore, implementing the proposed system will keep the cities free from hazardous diseases and environmental pollution by detecting the level of waste in the dustbins and the dumping grounds by providing a graphical image. We used an android application for locating the shortest path of reaching over one dustbin and generating alerts.

If we stick to the usual road map, then it might be the case when some half-filled dustbins would be cleaned first, whereas filled dustbins might get cleaned later [41, 42]. Then there will be overflowing of dustbins on the roads, which can lead to land pollution. The truck driver will be guided via a mobile application, which shows the priority of one dustbin over the other with the data stored via image processing. The tracking of waste collection trucks will provide an optimized route based on real-time data of waste levels in each city's waste collection site. The real-time sensor data will help find the priority of one dustbin over other bins, which can be synchronized with Google Map API and direct the truck driver along the best route from a high-priority location to a lower one. The proposed solution will avoid the overflow of any dustbin and reduce the unhygienic conditions in the city. Further, this technique would be helpful in the optimization of logistics as well as human resources by municipal agencies of cities.

Data used for this experimental setup are available at https://drive.google.com/file/d/1lE4GZq-sUzFsilIcGVgVScb87aorKJfW/view?usp=drivesdk.

### 5.1. Hardware

#### 5.1.1. Arduino UNO Microcontroller

Arduino UNO shown in Figure 5 is an ATmega328P-based microcontroller board (datasheet). It features 14 digital pins (including 6 PWM outputs), 6 analog inputs, a ceramic 16 MHz (CSTCE16M0V53-R0) resonator, a USB connection, power connector, an ICSP header, and a reset button. It has all the necessary elements to support the microcontroller; just connect it to a computer with a USB cable or power it to start using an AC-to-DC converter or battery. You can play with your UNO with no worries, and you can change the chip for a couple of bucks without thinking too much about doing something wrong.

#### 5.1.2. Ultrasonic Sensor

The ultrasonic sensor in Figure 6 is measuring equipment with ultrasonic sonic waves, which calculates the distance from an object. An ultrasonic sensor utilizes an ultrasonic pulses transducer to send out and receive information about the vicinity of an item. High-frequency sound waves reflect boundaries that generate different echo patterns.

#### 5.1.3. Moisture Sensor

This sensor shown in Figure 7 detects the volumetric content of water inside the soil and produces the level of wetness. The sensor is provided with analog and digital output, allowing for analog and digital usage. We will interface the sensor in this post in both modes. So let us start our lesson on the Arduino connecting moisture sensors with the soil.

#### 5.1.4. Buzzer

The piezo buzzer is also known as an Arduino buzzer shown in Figure 8. It is essentially a little speaker that you can link to Arduino directly. At a frequency, you may make it sound. The buzzer makes a sound on the back of the piezoelectric effect.

#### 5.1.5. LED

LEDs shown in Figure 9 are tiny, bright lights used for various purposes. To begin with, we will be working to blink a microscope LED, the Hello World. It is so basic that you switch on and off a light. Setting up this key basis is a strong foundation for you as we work on increasingly complicated tests.

#### 5.1.6. Jumper Wires

Cable Dupont is also known as jumper wires. They are cheap and useful for connecting devices like sensors, Arduino boards, and boards. The cable comprises the men to men, the men to women, and the women to men.

The two gadgets you wish to interconnect can be purchased from you. The Dupont cable is suitable for the inner wiring, the electronic project, and the genuine Arduino product in office equipment, audio, and video machines. They are robust, reusable, and easy to use and install.

## 6. Result Analysis

The proposed system architecture is shown in Figure 10. The smart dustbin is installed with an ultrasonic sensor that measures the dustbin's distance or level with ultrasonic waves and a moisture sensor, which detects whether the waste is wet or dry. The ultrasonic sensor and moisture sensor are connected to the Arduino UNO microcontroller unit. Power supply, LED, and buzzer are used in the above system. The data are sent to the receiver on the sender side on how many dustbin levels have been filled using IoT. On the receiver side, the user gets an indication through a mobile application.

According to the indications he received, he can notice how much of the dustbin level has filled. The proposed system does the following:

1. Identifying the filled dustbins
2. Indication of the system
3. Communication through IoT framework

The implementation of the system discussed above provides the optimized path for efficient waste collection. This system reduces infrastructure, rating, and maintenance costs by up to 30%. Smart bins outperform in comparison to ordinary garbage cans. It happens due to the amalgamation of digital waste monitoring and trash compaction technologies. In this way, a decrease up to 80% in the number of waste pickups is required, resulting in reduced labor, pollution, fuel use, and traffic congestion. Smart waste technologies are becoming more valuable, and they will continue to play a larger role in assisting private businesses and government agencies in improving efficiencies and meeting waste reduction targets.

The system proposed by the authors also eliminates the risk of unnecessary waste collection, including fuel and staff time. Waste generation rates are increasing around the globe. With rapid population growth, the amount of waste generated is expected to rise to 2.5 billion tons by 2026. According to a report on solid waste management by the United Nations, waste is an essential factor responsible for greenhouse gas emissions.  Figure 11 shows different kinds of waste which are generated at home.

## 7. Comparison with Other Systems

### 7.1. Integrated Linear Model (ILM)

ILM is a rectilinear model that decreases the overall price of solid waste in the community. An integrated linear model is a model that is used to reduce waste in the metropolitan city. This model is a balanced network model that is used for managing waste across the country. This model has three components:

1. Garbage-producing sector
2. Garbage-cleaning sector
3. Garbage-extracting greenhouse gases

Here, produced waste is handled by the waste cleaning sector, and the final waste is produced after recycling and altering into reusable elements. After conversion, it will be transferred to society.

### 7.2. Advanced Locality Model (ALM)

The main principle of the given model concentrates on the issue of managing waste in an environment-friendly manner. ALM can be controlled with the active contribution or participation of the good natives and enhance the nation's standard of living. The primary fundamental of the ALM is “Self Governance.”

### 7.3. Mixed-Integer Goal Programming Linear Model

The objective of this programming model is to obtain the initial matrix using the deviational variables as slacks. They also established the dual complication and displayed that the dual-based evaluation generates an absolute scale for the precedence element [43]. The expression of the mixed-integer goal programming model is constructed in pairs of primal and dual complications. The main aim of the given model is as follows:

1. Reverse administration rates
2. Extraneous wastepaper goal
3. Waste retrieval goal

### 7.4. Integer Programming Model (IPM)

This model is for an integrated arrangement of solid waste management. There are 77 quarters and eight separate quarters. This model aims to build a fertilizer plant, recycling system, automatic compost plant, Resource Description Framework (RDF) system, vermicular compost system, and the landfill area's development close by such a plant, decreasing transportation cost.

All the models mentioned above are based on some old technologies, and the model proposed by us is based on the latest technologies that are IoT (Internet of Things), ML (Machine Learning), GPS (Global Positioning System), and neural networks. A dumper truck database has been generated in the given system so that data and details of dumper truck ID, meeting date, meeting time of garbage collection, and so on are collected. This technique keeps track of all the truck driver's activities and the waste gathering system of waste management [17]. This system allows on-time waste gathering and allows automobile trace through database making use of GPS automation and decreases the drawback, such as usage of the minimal way, fuel price, cleansed nature, and available vehicle. The latest technologies and processes used in the above system are good enough to ensure practical consequences and a perfect green environment.

### 7.5. Comparison of Accuracy of Different Machine Learning Algorithms

The performance of a machine learning model can be improved by using a larger dataset. Scikit-learn offers four frequently used machine learning models. Random forest classifier is the initial model. A huge number of distinct samples of data are taken and “trees” are grown out of them. Based on the Bayes theorem and the assumption of independent predictors, the second model is a Naive Bayes classifier. As a kind of neural network, the third model considered is multilayer perceptron classifier. Hierarchical network architectures include input layers that enter input values into the network, layers that conduct feature categorization but hide findings, and layers that operate similarly to the hidden levels but reveal the results of the classification. The fourth model is support vector machine (SVM), which is used for binary classification. If a new data point arrives on one side of a hyperplane, it may be classified. To train the four models, the pictures were tagged according to the type of waste and uploaded to a website. As a result of the scanning procedure, certain characteristics of the pictures were retrieved to be utilized in training and testing the model. Thus, the four models were trained to recognize 15,000 pictures of both biodegradable and nonbiodegradable garbage. The mean accuracy and the percentage accuracy obtained are shown in Table 1.

## 8. Conclusion

Using the Internet of Things, this study illustrates how smart waste management may be done. This method ensures that waste is collected as soon as it reaches the maximum level. As a result, the system will provide accurate reports, therefore boosting its efficiency. The authors intend to evolve a smart waste management system based on the perception of sustainable, integrated waste management. The closure of landfills could pose various potential hazards due to which public health may get affected. Open junkyards and the burning of undesirable wastes can lead to environmental pollution and many hazardous diseases. There should be a system that can effectively supervise the disposal and collection of waste and regulate the comprehensive growth of superfluous waste. The system proposed by us collects and efficiently treats the waste as compared to other models. It also saves fuel costs as well as time. The system is also tracking the garbage collecting trucks, which provides real-time trucks' real-time positions, thereby increasing work efficiency. All the previous waste management models mainly focus on increasing sustainability and ignoring the overall system's time and cost. However, our waste management technique is sustainable and reduces the time and cost of the setup. With the help of image processing, the system predicted the waste index of a particular dumping ground. According to the priority, the waste-collecting vans will collect waste, which saves much time. With respect to the infrastructure in India, the model proposed in this paper is designed to integrate the different stakeholders of the waste management system, such as smart bins and sensors at the source area and vehicles. The system is efficient and effective because smart bins, collection vehicles, and routes are dynamically updated.

## Figures and Tables

**Figure 1:** Waste management hierarchy.

**Figure 2:** Flowchart for smart waste management.

**Figure 3:** Real-time monitoring system.

**Figure 4:** Experimental setup.

**Figure 5:** Arduino UNO microcontroller.

**Figure 6:** Ultrasonic sensor.

**Figure 7:** Moisture sensor.

**Figure 8:** Buzzer.

**Figure 9:** LED.

**Figure 10:** Flow graph of Arduino UNO.

**Figure 11:** Graph showing different types of waste generated.

**Table 1:** Comparison of the accuracy of the four models.

Algorithm	Potential distribution modeling (%)	Mean accuracy	Percentage accuracy (%)
Support vector machine	87.23	0.8951	89.51
Random forest classifier	91.43	0.9749	97.49
Multilayer perceptron	N/A	0.9644	96.44
Naive Bayes	84.14	0.8146	81.46

## Data Availability

The data used to support the findings of this study have been deposited in the https://drive.google.com/file/d/1lE4GZqsUzFsilIcGVgVScb87aorKJfW/view?usp=drivesdk repository. Coding is available for this article whenever required.
